This article has been retracted.

# The Role of Gender-Related Immune Genes in Childhood Acute Myeloid Leukemia

**DOI:** 10.1155/2022/3235238

**Published:** 2022-09-23

**Authors:** Lu Hao, Qiuyan Chen, Xi Chen, Qing Zhou

**Affiliations:** ^1^Science and Education Department, Shenzhen Baoan Shiyan People's Hospital, Shenzhen, China; ^2^Central Laboratory, The People's Hospital of Baoan Shenzhen, The Second Affiliated Hospital of Shenzhen University, Shenzhen, China

## Abstract

The study of immune genes and immune cells is highly focused in recent years. To find immunological genes with prognostic value, the current study examines childhood acute myeloid leukemia according to gender. The TARGET database was used to gather the “mRNA expression profile data” and relevant clinical data of children with AML. To normalize processing and find differentially expressed genes (DEG) between male and female subgroups, the limma software package is utilized. We identified prognostic-related genes and built models using LASSO, multivariate Cox, and univariate Cox analysis. The prognostic significance of prognostic genes was then examined through the processing of survival analysis and risk score (RS) calculation. We investigated the connections between immune cells and prognostic genes as well as the connections between prognostic genes and medications. Finally, five immune genes from the TARGET database have been identified. These immune genes are considerably correlated to the prognosis of male patients.

## 1. Introduction

One of the most frequent blood malignancies, acute myeloid leukemia (AML), makes up about 1% of all cancers [1–4]. Because of the clonal growth of “undifferentiated myeloid progenitor cells,” reduced haematological function and failed bone marrow (BM) are characteristics of AML, both of which can have fatal consequences [5–7]. The main treatment strategy of AML was intensive induction chemotherapy and postremission treatment. Although many AML patients can obtain significant remission through chemotherapy at first, the complete elimination of the disease is still rare and it is very easy to relapse. Pediatric AML accounts for about 25% of pediatric leukemia. Although the incidence is relatively low, the prognosis is poor, so it has a very huge clinical challenge [8–11]. Pediatric AML is a complex disease. The response to treatment varies greatly, even in tumors with comparable histological features. Therefore, we are interested in learning how men and women differ in children AML.

The “tumor microenvironment” (TME) has collected a lot of interest recently [12–15] due to its potential significance in the growth of cancer. TME indicates the cellular setting in which tumor lesions are present. The two most important nontumor components among them, stromal cells and immune cells, were of key significance to the diagnosis and prognosis of cancer [16–20]. Our knowledge of the immunological microenvironment's function is still lacking, nevertheless, because of its complexity and dynamic nature. Immune cells that have infiltrated tumors were a part of a complex microenvironment [21–23]. Strengthening research on tumor immune cell infiltration in children with AML was particularly important. They are crucial in preventing or promoting the growth and development of tumors. We can develop and use these effects to study the effective targeting of drugs and improve the prognostic survival of patients.

For this work, we used clinical data from the TARGET database to match the “mRNA expression profile data” of children having AML. In order to study the difference in gender in children AML, we performed differential genetic identification between the male subgroup and the female subgroup. To discover the function and role of immune genes, we screened immune-related genes from DEGs. GO and KEGG analysis results show that it is related to some important functional pathways in tumors. The prognosis-related genes are screened to evaluate the prognostic significance of important genes. The association and relationship between important genes and immune cells was examined using the “CIBERSORT algorithm” to assess the immune cell situation of the male subgroup.

We further explored the association of key genes and drugs.

## 2. Materials and Methods

### 2.1. Database

Children with AML have their mRNA expression reports and accompanying clinical data gathered from TARGET [24]. Clinically insufficient data was removed and classified by gender. In the male group, there were 186 patients, and in the female group, there were 172 patients.

### 2.2. Detection of Gender-Related Immune Genes

Using the “limma package,” various stated genes (DEGs) were discovered between the male and female groups [25, 26]. Adjusted *p* value < 0.05 and genes with |log FC| > 1 were defined as DEGs. ImmPort database [27] was used to obtain immune-related gene sets. Then, we screened the immune genes in DEGs and visualized them through an online website [28].

### 2.3. Analysis of DEGs

The database Kyoto Encyclopedia of Genes and Genomes (KEGG) is utilized in deducing advanced role of biological systems from molecular-level information. Gene Ontology (GO) can be utilized to carry out enrichment analysis. We used “org.Hs.eg.db,” “clusterProfiler,” “richplot,” and “ggplot2” software packages to carry out KEGG and GO function enrichment analyses on DEGs. A *p* < 0.05 was set as a “cut-off criterion.”

### 2.4. Survival Analysis and Cox Regression and ROC Curve

A univariate Cox analysis was performed on the identified key DEGs, and a *p* of <0.05 was considered meaningful. To identify the most important prognostic genes, the LASSO analysis and multivariate Cox were carried out in both gender groups, respectively. A model was then built. The “LASSO coefficients” (*β*) observes the following: Risk Score =∑_*i*=1_^*n*^Expi *βi* [29–31].

In the above formula, the *βi* stands for the regression coefficient, while Exp shows the gene expression value. By comparing specificity and sensitivity of risk-based survival prediction, using OS time (1, 3, and 5 years) of the patient, “ROC” curves are used to assess prognostic performance accuracy. In order to evaluate the prognostic value, the part under the curve (AUC) was also determined.

### 2.5. Evaluation of Immune Cell Type Fractions

A potent analytic technique called CIBERSORT uses gene expression profiles made up of 547 genes [32–34]. It precisely quantifies the components of various immune cells. It employs a deconvolution technique to distinguish each type of immune cell. We subsequently examined the immune cell infiltration in male subsection using the results of the prior investigation. The maximum limit established was at *p* value (0.05).

### 2.6. The Correlation Analysis between Key Genes and Drugs

In the current research, the R software is applied to examine the main gene-drug interactions in our work after acquiring data on gene-drug interactions from the CellMiner database [35].

### 2.7. Analysis

The “glmnet” software programme was used to conduct the LASSO analysis. To plot the survival ROC, we used the “survivalROC” software tool. The “rmda” software package was used to do the decision curve analysis. The “nomogram” and “calibration” diagrams have been created by using the “rms” software package. The “survival” software package is utilized to calculate the c-index and conduct a survival analysis. R version 3.5.1 was employed to conduct the aforementioned investigation, and “*p* 0.05” was thought as an important value.

## 3. Result

### 3.1. The Identification of Differentially Expressed Gender-Related Prognostic Immune Genes and Functional Enrichment Analysis in Children AML

We separated the mRNA expression data for children's AML into subgroups of males and females using the TARGET database, and then, we looked for differences in the genes between the two. According to the findings, there were 118 DEGs that were notably upregulated, while 286 DEGs were downregulated (Figure 1(a)). First 50 genes were visualized (Figure 1(b)). Then, we compared DEGs with the immune gene set to obtain immune-related DEGs (*n* = 57). Then, GO and KEGG enrichment evaluation took place (Table 1) using R software (Figures 1(c)–1(e)).

### 3.2. Model Construction and Verification

Male and female subgroups were imperiled to “univariate Cox analysis,” where results revealed that 10 genes in the male subgroup and 4 genes in the female subgroup were significantly related to prognosis (Table 2). Then, to screen genes, we used LASSO analysis. The female subgroup's outcome was 0, which has no analytical significance (Figures 2(c) and 2(d)). The male subgroup's outcome was significant (Figures 2(a) and 2(b)). Then, a multifactor Cox analysis on the male subgroup was further performed, and 5 genes (MET, MMP9, MUC4, SEMA3D, and TSLP) used to construct the model were identified (Table 3). For the prognostic ability evaluation of a given standard, we divided male subgroups. The median risk score was the base for this subgroup. Patients were categorized into high-risk and low-risk groups. Patients' survival was then analyzed. The findings demonstrated that the OS rate of the group having more risk decreased as compared to one having low risk (Figure 2(e)). The assessment can be performed in better way by the prognosis of this model by completing the time-related ROC analysis (Figure 2(f)). Additionally, the “survival status distribution,” “risk score distribution,” and “heat map” were examined (Figures 2(g)–2(i)). WT1 mutation and risk score can be employed as independent prognostic indicators for the model as per the findings of univariate and multivariate Cox analysis (Figure 3). In addition, we used 5 genes including MET, MMP9, MUC4, SEMA3D, and TSLP to construct nomograms to foresee one-, three-, and five-year OS (Figure 4(a)). We also constructed a calibration graph. Good accord was observed between the expected and observed findings as shown by graph below (Figures 4(b)–4(d)).

### 3.3. The Relationship between Genes of the Model and Immune Infiltrating Cells

CIBERSORT was employed for evaluation of 22 immune cells in man patients (Figure 5(a)). A heat map is created (Figure 5(b)), as well as analyzed the association of various “immune infiltrating cells.” The objective was to discover relationship between “immune infiltrating cells” in the male subgroup and genes of the model (Figure 5(c)). A high immune cell score is linked to a poor prognosis, according to the results of a survival analysis, later on we conducted (*p* = 0.034; Figure 6(a)). Furthermore, we looked at the association and relationship between prognosis and the expression levels of various immune cells. The results revealed that high expression of T cells CD4 naive (*p* = 0.002), macrophage M1 (*p* = 0.032), and T cell gamma delta (*p* 0.001) was associated with a reduced and poor prognosis, whereas high expression of B cells naive (*p* = 0.025) was associated with a better prognosis (Figures 6(b)–6(e)). Finally, the connection between genes and immune cells was examined, and *p* < 0.05 was considered meaningful (Figures 6(f)–6(i)). The results showed that MET has a positive relationship with macrophage M1 (*R* = 0.36, *p* = 2.2e − 05), MUC4 consumes an encouraging association with T cell follicular helper (*R* = 0.74, *p* < 2.2e − 16), MMP9 and macrophage M0 interact favorably (*R* = 0.82, *p* < 2.2e − 16), and SEMA3D has a positive relationship with mast cells activated (*R* = 0.4, *p* = 1.9e − 06).

### 3.4. The Correlation between Drugs and Genes

We examined the association between the model's genes and medications in order to further examine their potential relevance in clinical treatment, and we then displayed the top 16 with the highest correlation (Figure 7). The results show that *MUC4* has a negative relationship with pelitrexol (Cor = −0.613, *p* < 0.001), epothilone B (Cor = −0.610, *p* < 0.001), and floxuridine (Cor = −0.438, *p* < 0.001). *MMP9* has a helpful relationship with rebimastat (Cor = 0.559, *p* < 0.001). *MET* has a negative association with lomustine (Cor = −0.532, *p* < 0.001), fenretinide (Cor = −0.472, *p* < 0.001), lmexon (Cor = −0.466, *p* < 0.001), carmustine (Cor = −0.464, *p* < 0.001), and XK-469 (Cor = −0.456, *p* < 0.001) and a positive correlation with staurosporine (Cor = 0.491, *p* < 0.001) and kahalide f (Cor = 0.437, *p* < 0.001). *SEMA3D* has a positive correlation with E-7820 (Cor = 0.527, *p* < 0.001) and a positive association with mithramycin (Cor = −0.518, *p* < 0.001) and depsipeptide (Cor = −0.470, *p* < 0.001).

## 4. Discussion

Due to the rapid advancement of immune checkpoint treatment in recent years such as CTLA-4 and PD-1 in AML, scientists have paid more and more attention to the research of immune genes and immune cells [36–40]. About 25% of paediatric leukemia is paediatric AML. Although the incidence is relatively low, the prognosis is poor, so it has a very huge clinical challenge. In addition, childhood leukemia also has great heterogeneity between tumors, so we want to explore the difference between male and female leukemia. This research used TARGET database to get the “mRNA expression profile data” of children with AML and the related clinical data. Gender based male and female groups were made and differential genes were found in male and female groups which were *n* = 186 and *n* = 172, respectively. The outcome was that 118 DEGs were considerably upregulated and 286 DEGs were significantly downregulated (Figure 1(a)). Then, we screened out 57 immune-related genes (Figure 1(c)).

GO analysis results show that “cytokine receptor binding,” “cytokine activity,” “growth factor activity,” “growth factor receptor binding,” “chemokine receptor binding,” “chemokine activity,” “G protein-coupled receptor binding,” “transforming growth factor-beta receptor binding,” etc. have performed significant roles. KEGG analysis results show that many “cancer-related pathways” play a role in it. This may include “cytokine-cytokine receptor interaction,” “IL-17 signaling pathway,” “JAK-STAT signaling pathway,” “TNF signaling pathway,” “chemokine signaling pathway,” “transcriptional misregulation in cancer,” “MAPK signaling pathway,” and “PI3K-Akt signaling pathway.”

“Univariate Cox analysis” was conducted on these immune-related DEGs in order to further examine them. The findings revealed that 10 genes in the group of males and 4 genes in the group of females were associated with prognosis (Table 1). “LASSO analysis” and “multivariate Cox analysis” revealed 5 independent prognostic genes in the male group, but no genes were screened in the female group (Figures 2(a)–2(d)). Patients in male subgroup were divided into high- and low-risk groups on the basis of median risk score. Then, their survival rate was examined to assess the prognostic capability of this model. According to the findings, the high-risk subgroup patients had a considerable low OS rate than that of the low-risk subgroup (*p* = 0.014; as shown in Figure 2(e). Risk score can be utilized as an independent “prognostic indicator” for the model, according to the findings of “univariate and multivariate Cox analyses” (Figure 3). We also created a nomogram to forecast one-year, three-year, and five-year OS.

To analyze the formation and composition of 22 immune cells in male patients, we employed CIBERSORT in order to investigate the association between “immune infiltrating cells” in the male subgroup and model genes (Figure 5(a)). The results of survival analysis exhibited that high scores were associated to poor prognosis (*p* = 0.034; Figure 6(a)). The association and correlation results show that high expression of “T cell CD4 naive (*p* = 0.002),” “macrophage M1 (*p* = 0.032),” and “T cell gamma delta (*p* < 0.001)” was associated with a poor prognosis, and high expression of B cells naive (*p* = 0.025) was related to better prognosis (Figures 6(b)–6(e)). Additionally, the link between genes and immune cells showed that MET has a positive connection with “macrophage M1 (*R* = 0.36, *p* = 2.2e − 05),” *MUC4* has a positive relationship with “T cell follicular helper (*R* = 0.74, *p* < 2.2e − 16),” *MMP9* has a positive association with “macrophage M0 (*R* = 0.82, *p* < 2.2e − 16),” and *SEMA3D* has a positive relationship with “mast cells activated (*R* = 0.4, *p* = 1.9e − 06).”

The association between genes and drugs was also assessed. The results show that *MUC4* has a negative relationship with “pelitrexol (Cor = −0.613, *p* < 0.001),” “epothilone B (Cor = −0.610, *p* < 0.001),” and “floxuridine (Cor = −0.438, *p* < 0.001).” *MMP9* has a positive association with “rebimastat (Cor = 0.559, *p* < 0.001).” *MET* has a negative connection with “lomustine (Cor = −0.532, *p* < 0.001),” “fenretinide (Cor = −0.472, *p* < 0.001),” “lmexon (Cor = −0.466, *p* < 0.001),” “carmustine (Cor = −0.464, *p* < 0.001),” and “XK-469 (Cor = −0.456, *p* < 0.001)” and a positive relationship with “staurosporine (Cor = 0.491, *p* < 0.001)” and “kahalide f (Cor = 0.437, *p* < 0.001).” *SEMA3D* has a positive connection with “E-7820 (Cor = 0.527, *p* < 0.001),” “mithramycin (Cor = −0.518, *p* < 0.001),” and “depsipeptide (Cor = −0.470, *p* < 0.001).”

One of the widely studied matrices is “metalloproteinases (MMPs).” MMP-9 is a key protease that is essential for numerous biological processes and can be utilized as a range of cancer biomarkers, according to previous research findings [41, 42]. A possible therapeutic target for several cancers (non-small-cell lung cancer) is the hepatocyte growth factor receptor (MET) (NSCLC). Numerous mechanisms that impact the survival, proliferation, and invasiveness of cancer cells are thought to be involved in the activation of the MET pathway in NSCLC [43]. Being a membrane-bound mucin, MUC4 accelerates the growth of different carcinomas. It is frequently suggested as a “promising biomarker” [44–46]. In pancreatic cancer immunotherapy, MUC4 has become a new tumor antigen. A secreted protein called SEMA3D has been associated with the happening and development of thyroid, pancreatic, and colorectal cancers [47, 48]. Thymus stromal lymphopoietin (TSLP) is a key cytokine for Th2 immunity. It has been proven that TSLP is believed as an important element to keep up immune homeostasis and adjust mucosal barrier inflammation. It plays a key role in inflammatory diseases and cancer [49, 50].

## 5. Conclusion

The results show the 404 differential genes from the male and female subgroups. In the Venn diagram, 57 intersect genes related to immunity were screened. “Functional enrichment cluster analysis” revealed the potential role of intersecting genes. Through “univariate Cox analysis,” “multivariate Cox analysis,” and “LASSO analysis,” five prognostic-related genes were identified in the male subgroup. RS was calculated. The findings of “survival analysis” exhibited that high RS was linked to a reduced and poor overall survival (*p* = 0.014). The results show that these 5 genes have good predictive power. We evaluated the immune cell scores in the male subgroup through the CIBERSORT algorithm showing that high scores were related to a reduced and poor prognosis (*p* = 0.034). We also found that prognostic genes were related to some “immune infiltrating cells.” We have identified 5 immune genes from the TARGET database that has an important relationship with the prognosis of male patients.

Through this research, we provide new approach to assess the function of gender-related immune genes in AML, especially in the male subgroup. In addition, the results may provide us with new prognostic indicators and help in future treatment.

In future work, in this study, we revisited the role of 5 genes in childhood AML, especially in the male subgroup. These results may help the study of AML in children. However, there are some limitations and drawbacks of this research. At first, research data mainly comes from the TARGET database. Most patients are Asian or from white race. Therefore, we should be extra cautious when extending the results of the study to patients who do not belong to the above mention races. Second, the consistency of the findings of the study lacks “in vitro or in vivo experiments.”

Overall, the role of gender-related immune genes in the prognosis of childhood leukemia is thoroughly investigated.

## Figures and Tables

**Figure 1:** Identification of differentially expressed gender-related prognostic immune genes and functional enrichment analysis in children AML. (a, b) Identification of DEGs in male and female subgroups. (c) Identification of immune-related DEGs. (d, e) GO and KEGG analyses.

**Figure 2:** Model construction and verification. (a, b) LASSO analysis in male subgroup. (c, d) LASSO analysis in female subgroup. (e) Survival analysis according to risk score. (f) Time-dependent ROC analysis for 1-, 3-, and 5-year overall survival (OS) of a prognostic model. (g) Heat map. (h) The relationship among the risk score. (i) Survival status of patients in different groups.

**Figure 3:** Forest plot of the univariate (a) and multivariate (b) Cox regression analysis in the male pediatric cohort for acute myelogenous leukemia (AML).

**Figure 4:** Nomogram. (a) Nomogram to predict 1-, 3-, and 5-year OS. (b–d) Calibration plots of the nomogram.

**Figure 5:** The CIBERSORT to evaluate the composition of 22 immune cells in male patients.

**Figure 6:** The relationship between genes of the model and immune infiltrating cells. (a) Relationship between immune cell score and survival. (b–e) The relationship between expression levels of different immune cells and prognosis. (f–i) The correlation between genes and immune cells.

**Figure 7:** The relationship between genes and drugs (visualized the top 16 with the highest correlation).

**Table 1:** Result of evaluation.

	Description	*p* value	KEGG	Description	*p* value
BP	Response to lipopolysaccharide	2.35E-14	KEGG	Cytokine-cytokine receptor interaction	4.87E-20
BP	Response to molecule of bacterial origin	4.14E-14	KEGG	IL-17 signaling pathway	6.58E-09
BP	Cellular response to lipopolysaccharide	6.45E-13	KEGG	JAK-STAT signaling pathway	6.22E-08
BP	Cellular response to molecule of bacterial origin	9.61E-13	KEGG	Rheumatoid arthritis	1.15E-07
BP	Cellular response to biotic stimulus	3.42E-12	KEGG	Viral protein interaction with cytokine and cytokine receptor	2.03E-07
BP	Leukocyte chemotaxis	9.23E-10	KEGG	TNF signaling pathway	4.88E-07
BP	Cell chemotaxis	1.13E-09	KEGG	Legionellosis	2.98E-05
BP	Antimicrobial humoral response	7.96E-11	KEGG	Amoebiasis	4.50E-05
BP	Granulocyte chemotaxis	2.65E-09	KEGG	Chemokine signaling pathway	0.00021
BP	Antimicrobial humoral immune response mediated by antimicrobial peptide	1.82E-09	KEGG	Malaria	0.000285
CC	Collagen-containing extracellular matrix	1.58E-05	KEGG	Inflammatory bowel disease	0.000779
CC	Secretory granule lumen	2.95E-05	KEGG	Transcriptional misregulation in cancer	0.001381
CC	Cytoplasmic vesicle lumen	3.19E-05	KEGG	Pertussis	0.001402
CC	Vesicle lumen	3.32E-05	KEGG	EGFR tyrosine kinase inhibitor resistance	0.001618
CC	Golgi lumen	0.000188	KEGG	African trypanosomiasis	0.001685
CC	Tertiary granule lumen	0.000486	KEGG	Measles	0.001922
CC	Specific granule lumen	0.000691	KEGG	Phospholipase D signaling pathway	0.00253
CC	External side of plasma membrane	0.000767	KEGG	MAPK signaling pathway	0.002611
CC	Endoplasmic reticulum lumen	0.001677	KEGG	TGF-beta signaling pathway	0.00306
MF	Receptor ligand activity	1.38E-28	KEGG	Hematopoietic cell lineage	0.003689
MF	Signaling receptor activator activity	1.83E-28	KEGG	AGE-RAGE signaling pathway in diabetic complications	0.003824
MF	Cytokine activity	2.34E-23	KEGG	Chagas disease	0.004106
MF	Cytokine receptor binding	3.65E-21	KEGG	Toll-like receptor signaling pathway	0.004401
MF	Growth factor activity	6.99E-19	KEGG	Tuberculosis	0.005838
MF	Growth factor receptor binding	2.09E-10	KEGG	Axon guidance	0.005975
MF	Chemokine receptor binding	9.74E-10	KEGG	NOD-like receptor signaling pathway	0.005975
MF	Chemokine activity	6.83E-09	KEGG	PI3K-Akt signaling pathway	0.007218
MF	G protein-coupled receptor binding	1.32E-07	KEGG	Kaposi sarcoma-associated herpesvirus infection	0.0078
MF	Transforming growth factor beta receptor binding	1.61E-05	KEGG	Cortisol synthesis and secretion	0.008345
			KEGG	Osteoclast differentiation	0.009117

**Table 2:** Univariate Cox analysis results of male and female subgroups.

ID	HR	HR.95L	HR.95H	*p* value
Male				
CHIT1	1.000138	1.000015	1.000262	0.028135
CXCL1	1.000132	1.000004	1.00026	0.043748
CXCL13	1.000421	1.000072	1.00077	0.017917
FAM19A5	1.007364	1.001897	1.012861	0.008233
MET	1.000143	1.000018	1.000268	0.025249
MMP9	1.000027	1.000008	1.000045	0.005283
MUC4	1.000697	1.000217	1.001178	0.004437
PDGFA	1.000147	1.000017	1.000277	0.026806
SEMA3D	1.000669	1.000167	1.001172	0.008968
TSLP	1.002514	1.00034	1.004693	0.023424
Female				
EREG	1.000003	1	1.000005	0.034576
FGF10	1.001333	1.000475	1.002191	0.002324
IL1A	1.000305	1.000083	1.000527	0.007056
NR0B1	1.004578	1.000491	1.008682	0.028106

**Table 3:** Multivariate Cox analysis results.

ID	HR	HR.95L	HR.95H	*p* value
MET	1.000132	1.000007	1.000257	0.037817
MMP9	1.000022	1.000001	1.000044	0.039233
MUC4	1.000785	1.000291	1.001279	0.00185
SEMA3D	1.000555	1.000007	1.001104	0.047121
TSLP	1.003106	1.00091	1.005307	0.005552

## Data Availability

The datasets analyzed in the current study are available in the TARGET database (https://ocg.cancer.gov/programs/target/data-matrix).
